The article "The Construction of the Evaluation Index for the Outgoing Auditing of the Natural Resource Assets of Local Leading Cadres Based on the Analytic Hierarchy Process" was retracted in 2023. Reasons: signs of a paper mill; compromised peer review; unreliable results or conclusions.

# The Construction of the Evaluation Index for the Outgoing Auditing of the Natural Resource Assets of Local Leading Cadres Based on the Analytic Hierarchy Process

**DOI:** 10.1155/2022/1215842

**Published:** 2022-01-24

**Authors:** Jiali Xuan

**Affiliations:** College of Business, Hohai University, Nanjing, 210000 Jiangsu, China

## Abstract

As the foundation of human survival and development, natural resources affect every aspect of our lives, including life and health, financial security, and overall social security. This article describes building a system for valuing the assets of good NR in operation for local executives who employ analytic hierarchy process. Based on his bibliographic data, he has a deep understanding of the theoretical issues associated with the process of analytical hierarchy and the uncontrollable control of natural resource assets. In addition, he uses an analytic hierarchy process to create a system of metrics for the external management of local leaders' NR and analyzes examples through the newly established metrics system. As a result, the current mayor of this case is more than the responsibility of the previous mayor. During the period, natural and environmental conditions improved, especially in the areas of water and air resources, which are more relevant than they are today.

## 1. Introduction

After 30 years of reform and opening up, my country's economy has grown rapidly, many of which have been traded for excessive resource consumption and ecological destruction [1, 2]. Such measures have led to the deterioration of the natural environment, and Japan is currently growing from expanding growth, which increases input, to concentrated growth, which improves production efficiency and promotes sustainable and cooperative economic growth. We are changing the method [3, 4]. We will abandon natural resource management to promote ecological culture and encourage local leaders to consider comprehensive economic growth, the development and utilization of natural resources, and environmental and ecological protection in the process of governance. In accordance with the requirements of ecological construction, we will encourage the construction of a reasonable industrial structure and strengthen the development and utilization of nuclear power [5, 6]. Natural resource outbound assets are used to assess work and performance by local leadership, transforming a resource protection assessment system that focuses only on economic development rather than resource consumption into a sustainable and resource-friendly environmental performance and development evaluation system [7, 8].

Some researchers have found that the new natural resource management includes a small number of managers, low professional level, and unclear management responsibilities, and ecological reports say that there are major problems such as insufficient resource implementation and, from these perspectives, summarize and analyze existing problems [9]. Other researchers believe that pilot natural resource management programs should select areas where pilot management programs are implemented, with better ecological conditions and more serious ecological damage increase. This is still true at this stage of the implementation of NR [10]. Some scholars believe that local executives rarely precontrol the outward management of NR. If NR and the ecological environment are destroyed, recovery will take a long time. Managing the NR of extroverted local executives is a very important assessment system, as the goals of postmanagement ecological protection and sustainable development are difficult to achieve due to the large losses [11, 12].

The article "The Construction of the Evaluation Index for the Outgoing Auditing of the Natural Resource Assets of Local Leading Cadres Based on the Analytic Hierarchy Process" was retracted in 2023. Reasons: signs of a paper mill; compromised peer review; unreliable results or conclusions.

In summary, more attention is being paid to research on the transmission and management of natural resource assets. This is an important national rating system. However, there are still some issues in the process of managing the outflow management of natural resource assets. The problem is how to build the control indicator.

This paper first adopts the hierarchical analysis method to establish the valuation system of local executives' foreign natural resource asset management and analyzes the practical problems faced by local executives according to references. Analyze theoretical issues, and use analytic hierarchy processes to build a system of runoff control indicators for top local executives' natural resource assets. The newly established metric system is used to analyze case problems and draw relevant conclusions through the analysis.

## 2. Analytic Hierarchy Process and Research on Outgoing Audit of Natural Resource Assets

### 2.1. The Problems Existing in the Audit of the Departure of Natural Resource Assets of Local Leading Cadres

#### 2.1.1. The Barriers to Effective Access to Basic Data

NR are widely distributed throughout the country and are highly mobile. In addition, many resources have not yet been clearly investigated. Even if there is a physical quantity, it may be difficult to determine the actual data due to insufficient collection. Therefore, it is difficult to quantify resources. In addition to various methods of measuring the value of assets, the present value of future cash inflows can also be used for resources that can generate direct income. Estimated costs can be used for resources that cannot generate direct revenue. Due to its rarity, it is difficult to quantify its value in consideration of cost-effectiveness.

The article "The Construction of the Evaluation Index for the Outgoing Auditing of the Natural Resource Assets of Local Leading Cadres Based on the Analytic Hierarchy Process" was retracted in 2023. Reasons: signs of a paper mill; compromised peer review; unreliable results or conclusions.

#### 2.1.2. Difficulty of Ownership

The resources are widely distributed and may include rivers and mineral deposits, belonging to multiple states, and the boundaries are not clear, and it is difficult to determine the ownership. The development of NR often produces externalities such as water pollution and air pollution, and it is difficult to determine who is responsible. For example, in the smog in northern part of our country, it is difficult to judge whether it is the impact of coal or automobile exhaust. Some NR are mobile, and the production activities of one department affect another. For example, pollution in the lower reaches of a river may be caused by stocking in the upper reaches.

#### 2.1.3. Lack of National Accountability Mechanism

Due to the information asymmetry between the central and local governments, the central government has increased its investment in environmental governance, introduced relevant policies, built some ecological and cultural enterprises, and closed high-energy-consuming enterprises. But higher GDP growth will continue to bear the cost of environmental pollution and waste of resources. In our country's current financial system, senior managers may be punished due to environmental issues, but this is an exception and not very deterrent. There is an imbalance between local government's financial and environmental responsibilities. Due to the lack of environmental protection mechanisms, local governments will appear inactive on environmental issues, ignoring corporate pollution problems, leading to the destruction of NR, and it is the inaction of local governments that has become a protective symbol for enterprises. The lagging nature of the pollution problem and the division of responsibilities are difficult, often because of thunder and rain. Moreover, pollution is often a long-term problem, and it often takes years for waste of resources to show its drawbacks. The term of office of senior executives in our country is usually five years, and it is difficult to separate responsibilities.

### 2.2. The Basic Theory of Analytic Hierarchy Process

#### 2.2.1. Create a Hierarchical Model

Divide the decision-making objectives, and design the hierarchy according to the relationship between high-, medium-, and low-level factors (decision criteria) and the decision-making objectives [12]. The highest level is the purpose of the decision and the problem to be addressed. The lowest level refers to the best way to make a decision. Among these are the various factors and decision-making criteria that need to be considered most. For two adjacent layers, the top is called the target layer and the bottom is called the agent layer.

The article "The Construction of the Evaluation Index for the Outgoing Auditing of the Natural Resource Assets of Local Leading Cadres Based on the Analytic Hierarchy Process" was retracted in 2023. Reasons: signs of a paper mill; compromised peer review; unreliable results or conclusions.

#### 2.2.2. Create a Comparison Matrix (Pair Comparison)

When determining the weight between different levels of factors, it is often not easy to accept if it is just a quality result. Therefore, a permanent matrix method is used. That is, not all elements are compared together, and relatively scales are used to compare different properties with different elements and to reduce the difficulty of improving accuracy. For example, some standards compare shapes in pairs and classify them according to their importance.

## 3. Construction of the Evaluation Index for the Outgoing Audit of Local Leading Cadres' Natural Resource Assets Based on the Analytic Hierarchy Process

### 3.1. Analysis of Indicator Construction Ideas

NR and wealth management is a form of management created through relationships with resource and environmental representatives to meet the requirements of sustainable development and improve resource use and environmental efficiency. NR assessment is an important indicator for measuring the level of government leaders in fulfilling their obligations to manage NR assets and protect the ecological environment. The setting of valuation indicators for NR assets should be determined based on the clear purpose of the audit valuation, the scope of the valuation, and the content of the valuation. In order to determine these audit assessments, it is first necessary to identify the reasons for discontinuing the audit of NR assets.  Figure 1 shows the idea of building a pointer in this article.

### 3.2. The Content of the Outgoing Audit of NR Assets

Based on the SEEA-based environmental resource classification, this article mentions the “decisive” indicators that classify NR assets into six categories of water, land, ocean, forest, mineral, and air resources.

1. Water resources: water resources refer to water sources that can meet local water needs and are available or potentially available for a long time. Water resources, especially freshwater resources, are important and irreplaceable substances indispensable to life.
2. Land resource assets: when deciding whether a piece of land has asset characteristics, it must be managed in strict accordance with national laws and regulations. Only land that is currently in use or may be reused in the future can be recognized as land resources. Land resource assets defined in this way play an irreplaceable role in social development and have distinct material and economic characteristics.
3. Marine resources: the marine resources here not only are the organisms and various substances contained in the ocean but also include marine resources in a broad sense, such as the energy formed by the tides and the sediments that exist on the seafloor. Broadly speaking, the ocean is to provide leisure space to meet the entertainment needs of mankind and at the same time bring some economic benefits to mankind.
4. Forest resource assets: forest resources refer to not only trees but also the entire biological community, including the land where trees, forest animals, plants, and microorganisms inhabit. It exists in this range. Forests have the functions of purifying the air, conserving water sources, protecting the soil, and regulating the climate. They are essential resources for protecting and improving the living environment of human beings.
5. Mineral resources: mineral assets are resources with obvious economic value after long-term geological movement and action. Mineral resources are nonrenewable NR, which are nonrecyclable, nonrenewable, and easy to consume.
6. Air resources: atmospheric assets are gases and atmospheric-related substances that humans can use as energy sources or produce biological materials. Generally speaking, the most widely used atmospheric resources by mankind are wind energy and solar energy. The impact of climate has a major impact on people, brings people economic benefits, and harms people's economic benefits, but it is also an atmospheric resource. Every minute of human life is closely related to air resources, and changes in air resources have a huge impact on human health and living conditions.

The article "The Construction of the Evaluation Index for the Outgoing Auditing of the Natural Resource Assets of Local Leading Cadres Based on the Analytic Hierarchy Process" was retracted in 2023. Reasons: signs of a paper mill; compromised peer review; unreliable results or conclusions.

### 3.3. The Construction of NR Asset Outgoing Audit Evaluation Indicators

#### 3.3.1. Mineral Resource Management

The indicators of mineral resource management in this paper are the recovery rate of mineral resources, the total recovery rate of mineral resources, and the inventory and recovery rate of mineral resources.

#### 3.3.2. Atmospheric Resource Audit

In this article, the energy resource management indicators will be set as follows: comprehensive air quality index (API index), air quality improvement goals, good days, and heavy pollution days.

#### 3.3.3. Land Resource Management

This article defines land resource management indicators as follows: per capita arable land, percentage of completed arable land, land relocation capacity, water and soil adjustment, land use, and land desertification rate.

#### 3.3.4. Water Resource Management

This article stipulates that the water resource management indicators are as follows: total water supply, per capita water resources, total sewage treatment rate, cultivated land irrigation rate, average water output value, water quality change rate, water quality improvement target, water quality to level 3 assets water resources utilization rate, and protection rate (water quality is equal to or greater than level 3, which refers to the proportion of the main monitoring department water quality greater than level 3).

The article "The Construction of the Evaluation Index for the Outgoing Auditing of the Natural Resource Assets of Local Leading Cadres Based on the Analytic Hierarchy Process" was retracted in 2023. Reasons: signs of a paper mill; compromised peer review; unreliable results or conclusions.

#### 3.3.5. Forest Resource Management

This paper defines the forest resource management indicators as follows: increasing forest coverage rate, forest stock volume, annual growth rate, and forest reduction. Select the forest resources for your senior management tenure.

#### 3.3.6. Marine Resource Management

This paper takes the marine resource management index as a comprehensive seawater quality index, the concentration of pollutants entering the ocean, the marine sewage discharge rate, the marine industry efficiency, and the utilization and protection of marine resources.

On the basis of the above-mentioned research, a set of NR management index system for local officials was initially developed. The goal of this article is to establish an index system locally. Of course, an index system can also be designed according to the differences in the distribution of NRs and the unique resources and environmental characteristics of each region. This also makes the audit more substantive.  Table 1 shows the specific indicator system for the external management of NR assets by local leaders.

### 3.4. Modeling by Analytic Hierarchy Process

#### 3.4.1. Build a Hierarchical Structure Model Based on the Constructed NR Asset Outgoing Audit Evaluation Index System, as Shown in Figure 2

#### 3.4.2. Construct a Judgment Matrix

According to Satie's research, the focus of the analytic process of determining weights is to create a crisis table. The importance ratio of the two indicators at the measurement level is determined by expert scores. Use the 1-9 scale method to obtain the ratio of the importance of the two elements.  Table 2 shows the specific importance of scales 1-9.

#### 3.4.3. Hierarchical List Sorting and Its Consistency Check

However, in fact, when creating a pair comparison table, the above requirements cannot be met. Therefore, the matching table needs a certain degree of consistency. In other words, paired comparison tables can tolerate some inconsistencies.

Analysis shows that for a completely consistent comparison table, the characteristic value with the highest absolute value is equal to the dimension of the table. The consistency requirement of the comparison table is that the characteristic value with the highest absolute value is not much different from the dimension of the table.

To check the completeness of paired comparison *A*, calculate the measure-CI index of the inconsistency in comparison table *A* (*n* > 1 square table type).

(1) $$\begin{array}{c} \text{CI}=\frac{\lambda \left(A\right)-n}{n-1}, \end{array}$$

where 1 is the eigenvalue of the matrix *A* description.

The article "The Construction of the Evaluation Index for the Outgoing Auditing of the Natural Resource Assets of Local Leading Cadres Based on the Analytic Hierarchy Process" was retracted in 2023. Reasons: signs of a paper mill; compromised peer review; unreliable results or conclusions.

The RI procedure for determining the accuracy of comparison tables *A* can be found in the relevant data. RgI is called the Mean Randomized Consistency Index and deals with the determination of tables only. Calculate the random CR ratio compared to *A* based on the following formula.

(2) $$\begin{array}{c} \text{CR}=\frac{\text{CI}}{\text{RI}}. \end{array}$$

### 3.5. Comprehensive Evaluation Model

The NR asset rating of leading cadres is composed of qualitative indicators and quantitative indicators, and the final scoring uses a comprehensive scoring method. Score each indicator, weigh the indicator scores, and then multiply them to get scores for different asset management conditions. Weigh the scores of various NR asset managements, and finally get the sum of executives. The total score of the outgoing asset management valuation.

1. Evaluation method of quantitative index: the quantitative index is calculated by the auditor according to the specific value and converted into excellent, good, medium, and poor, giving 100, 80, 60, and 20 points, respectively.
2. Quality index evaluation method: for the quality index, the auditor evaluates the quality index, simply evaluates the final process, calculates the average value, and obtains the final score by setting the index to different scores of 100, 80, 60, and 20.

## 4. Instance Verification

Through the analysis of the actual situation of the audit of local leaders and local DBS assets, the above indicators are established to determine the appropriate valuation system. This paper uses an initiality comparison approach. Since the term of mayor is 2019 to 2020, this article compares the 2018 former mayor to the 2019 mayor score and compares the 2020 score. This result was used to assess the mayor's performance in the use of nurses and environmental protection responsibilities. According to the collected raw data, standardized processing is carried out.

The data is shown in Table 3.

According to the above calculation method, the comprehensive scores of the audit evaluation of the departure of NR assets during the term of the mayor of this city in 2018, 2019, and 2020 are obtained as shown in Table 4.

According to Figures 3 and 4, the total scores of NR-related assessments during the term of the current mayor are 79.53 points and 95.65 points, respectively. The final result of the comprehensive evaluation model is judged, and the scores are “good” and “excellent,” respectively, which are better than the previous recognition. During the term of the mayor, especially in the areas of water and air resources that are the most concerned today, NR and environmental conditions will be improved to ensure that public water safety and air pollution issues are properly resolved.

The article "The Construction of the Evaluation Index for the Outgoing Auditing of the Natural Resource Assets of Local Leading Cadres Based on the Analytic Hierarchy Process" was retracted in 2023. Reasons: signs of a paper mill; compromised peer review; unreliable results or conclusions.

## 5. Conclusions

In the early stage of China's social development, local administrators do not pay attention to the excessive consumption of natural resources and assets and are in a state of exchanging political results at the cost of damaging the ecological environment. To mitigate this side effect, the party and state have officially launched a natural resource asset valuation system to control overconsumption of natural resource assets. However, the management of NR for local leaders is still in the early stages of development, so some difficult problems are inevitably addressed in the actual process, limiting their implementation and promotion. It is inevitable.

After analyzing related theories, this paper studies the construction of NR assets out-of-service audit evaluation indicators for local leading cadres based on the analytic hierarchy process. Then examples were used to verify. The examples show that the comprehensive evaluation scores of NR assets during the tenure of the mayor are 79.53 points and 95.65 points, respectively, which are better than those of the previous mayor during his tenure.

## Figures and Tables

**Figure 1:** Framework diagram of indicator construction thinking analysis.

**Figure 2:** Hierarchical model diagram.

**Figure 3:** Original NR assessment score.

**Figure 4:** Comprehensive score of NR assets outgoing audit evaluation.

**Table 1:** Specific indicator system for external management of NR assets by local leaders.

Target layer A	Criterion level B	Evaluation layer C
Audit evaluation of the departure of NR assets of local leading cadres	Responsibility for implementing NR asset policy B1	NR policy implementation rate C11
		Compliance rate of NR policy C12
		NR policy adjustment rate C13
	Responsibility for the use of NR asset B2	NR fund disbursement rate C21
		NR fund utilization growth rate C22
		Social public satisfaction C23
	Liability for NR asset B3	Mineral resource C31
		Atmospheric resource C32
		Land resource C33
		Water C34
		Forestry resource C35
		Marine resource C36

**Table 2:** The importance of two-element scale.

Factor *i* vs. factor *j*	Scaling
Equally important	1
Slightly important	3
Stronger important	5
Strongly important	7
Extremely important	9
The middle value of two adjacent judgments	2, 4, 6, 8

**Table 3:** Original NR assessment score.

	2018	2019	2020
NR policy implementation rate C11	61.12	77.32	99.34
Compliance rate of NR policy C12	81.17	61.23	99.26
NR policy adjustment rate C13	61.02	99.21	87.23
NR fund disbursement rate C21	74.34	99.23	61.34
NR fund utilization growth rate C22	60.04	84.32	99.56
Social public satisfaction C23	60.06	77.21	99.67
Mineral resource C31	81.21	66.34	92.1
Atmospheric resource C32	61.02	72.56	99.48
Land resource C33	72.43	92.12	99.46
Water C34	73.41	75.78	84.32
Forestry resource C35	73.12	69.01	97.89
Marine resource C36	61.02	66.34	91.23

The article "The Construction of the Evaluation Index for the Outgoing Auditing of the Natural Resource Assets of Local Leading Cadres Based on the Analytic Hierarchy Process" was retracted in 2023. Reasons: signs of a paper mill; compromised peer review; unreliable results or conclusions.

**Table 4:** Comprehensive score of NR assets outgoing audit evaluation.

	2018	2019	2020
NR policy implementation rate C11	2.723	3.574	4.23
Compliance rate of NR policy C12	2.309	1.719	2.73
NR policy adjustment rate C13	6.534	10.82	9.25
NR fund disbursement rate C21	2.723	3.51	2.176
NR fund utilization growth rate C22	3.412	4.873	5.67
Social public satisfaction C23	8.226	10.564	13.45
Mineral resource C31	4.517	3.552	4.647
Atmospheric resource C32	9.742	1.715	16.21
Land resource C33	5.937	10.82	8.01
Water C34	13.012	3.53	17.42
Forestry resource C35	7.836	4.872	10.62
Marine resource C36	4.521	3.521	4.631

## Data Availability

The data underlying the results presented in the study are available within the manuscript.
